The article "Lessons From Recurrent Dropped Head Syndrome After Inadequate Short Fixation: A Case Series" was published in 2025. Journal: Cureus.

# Lessons From Recurrent Dropped Head Syndrome After Inadequate Short Fixation: A Case Series

**DOI:** 10.7759/cureus.86041

**Published:** 2025-06-15

**Authors:** Eiichiro Honda, Tatsuya Tanaka, Xuan Liu, Keishi Tsunoda

**Affiliations:** 1 Department of Neurosurgery, Shiroishi Kyoritsu Hospital, Shiroishi, JPN; 2 Department of Neurosurgery, International University of Health and Welfare Narita Hospital, Narita, JPN; 3 Department of Spinal Surgery, Kawasaki Hospital, Yame, JPN

**Keywords:** activities of daily living, cervical kyphosis, cervical sagittal alignment, corrective spinal fusion, dropped head syndrome, isolated neck extensor myopathy, long-segment fixation, sagittal vertical axis

## Abstract

Dropped head syndrome (DHS) is a condition in which the head falls forward due to dysfunction or atrophy of the cervical extensor muscles. It is more commonly observed in elderly women and significantly affects horizontal gaze and activities of daily living (ADL). For cases in which conservative treatment is ineffective, surgical corrective fixation is considered; however, indications and standardized procedures have not yet been fully established.

We retrospectively analyzed five cases of DHS treated surgically at our institution and examined the efficacy of corrective fixation and potential treatment strategies. Five patients (mean age: 82.6 years; all female) who underwent surgery for DHS between 2018 and 2024 were included. Three patients initially underwent short-segment fixation or laminoplasty, but DHS recurred. Eventually, all cases required long-segment fixation extending from C2 or the occiput to Th1/Th2.

Radiological evaluations included measurements of the C2-C7 Cobb angles, sagittal vertical axis (SVA), and T1 slope before and after surgery. All patients exhibited cervical kyphosis and sagittal imbalance. Postoperatively, cervical lordosis was restored, and improvements were noted in SVA and T1 slope. In four cases, patients were able to maintain horizontal gaze for over 30 minutes, and improvements in ADL living were observed. One patient died from aspiration pneumonia, although horizontal gaze was maintained postoperatively.

Long-segment corrective fixation within an appropriate range is considered a safe and effective treatment option.

## Introduction

Dropped head syndrome (DHS) is a condition characterized by severe flexion of the head due to weakness and atrophy of the cervical extensor muscles, significantly impairing activities of daily living (ADL) [1-6]. It predominantly affects elderly women and may be accompanied by difficulty maintaining a horizontal gaze and neck pain; in advanced cases, dysphagia and gait disturbance can also occur [3, 4, 6, 7]. The etiology of DHS is diverse and includes isolated neck extensor myopathy (INEM), age-related cervical spondylotic changes, and neurodegenerative disorders such as Parkinson’s disease and amyotrophic lateral sclerosis [2, 4, 6-8]. Additionally, cervical kyphosis, spondylolisthesis, and sagittal malalignment are believed to contribute to disease progression [5, 6, 9, 10]. Although conservative treatment with rehabilitation and orthotic support is typically the first-line approach, surgical correction and fixation may be considered for progressive cases or those refractory to non-operative measures [3, 4, 6, 8, 10, 11]. In particular, in cases with flexible and reversible kyphotic deformities, selecting an appropriate fusion range can lead to favorable sagittal realignment and functional improvement [6, 10-12].

In this report, we retrospectively reviewed five patients who underwent surgical treatment for DHS at our institution between 2018 and 2024. We discuss the radiographic findings, surgical techniques, and postoperative outcomes, focusing on the efficacy of corrective fixation and treatment strategy for DHS.

## Case presentation

We retrospectively reviewed five patients with DHS who underwent surgical treatment at our institution between 2018 and 2024 (Table 1). All patients were female, with a mean age of 82.6 years (range: 69-91 years).

**Table 1:** Summary of surgical cases with dropped head syndrome C: cervical; T: thoracic; O: occipital; SVA: sagittal vertical axis; +: kyphosis is present Note: The numerical identifiers (e.g., Case 1, Case 2, Case 3, etc.) used in the table are arbitrary and were created solely for the purpose of referencing specific cases within this article. These identifiers do not correspond to any patient-identifying information.

Case	Age (years)	Sex	Dropped head symptoms onset type	Other symptoms	Kyphosis	Preope			Surgical method	Postope		Result
						C2-C7 Cobb angle (°)	C2-C7 SVA (mm)	T1 slope (°)		C2-C7 SVA (mm)	T1 slope (°)	
1	69	Female	Acute (days)	Radiculopathy	+	-42	35.5	11	C4–C6 anterior-posterior fusion→O–T2 posterior fusion	21.7	6	Improvement
2	89	Female	Slow onset (months)	Myelopathy	+	-7	37.5	20	Laminoplasty→C2–T1 posterior fusion	11.2	12	Improvement
3	91	Female	Slow onset (months)	Myelopathy	+	-3	41	43	C2–T2 posterior fusion	18.2	27	Died of pneumonia
4	83	Female	Slow onset (months)	Radiculopathy	+	-21	70.7	27	C2–T1 posterior fusion	30.1	14	Improvement
5	81	Female	Slow onset (months)	Radiculopathy	+	-49	32	24	C5–C7 anterior-posterior fusion→C2–T1 posterior fusion	-5	8	Improvement

One patient (Case 1) presented with an acute-onset type, characterized by a sudden inability to maintain horizontal gaze. The remaining four patients (Cases 2-5) exhibited a gradually progressive type over several months. Myelopathy was observed in two cases (Cases 2 and 3), while radiculopathy was present in three cases (Cases 1, 4, and 5). Plain radiographs demonstrated evident cervical kyphosis in all patients (Figure 1).

**Figure 1:** Preoperative neutral lateral cervical radiographs A: Case 1; B: Case 2; C: Case 3; D: Case 4; E: Case 5. Lateral cervical radiograph demonstrating kyphosis. The curvature is emphasized using a red curved line to illustrate the abnormal alignment. The numerical identifiers (e.g., Case 1, Case 2, Case 3, etc.) are arbitrary and were created solely for the purpose of referencing specific cases within this article. These identifiers do not correspond to any patient-identifying information.

The C2-C7 Cobb angle ranged from −3° to −49° (normal range: 20° to 40° lordosis), indicating pathological kyphotic alignment. The sagittal vertical axis (SVA) at C2-C7 ranged from 32 to 70.7 mm (normal range: 10-40 mm), suggesting anterior displacement of the cervical spine. The T1 slope ranged from 11° to 43° (normal range: 13° to s25°), with many cases showing abnormally elevated values, reflecting sagittal imbalance. In Cases 2 and 3, T2-weighted MRI revealed spinal canal stenosis and high-signal intramedullary changes.

Initial surgery included laminoplasty and/or short-segment posterior fusion in three cases (Cases 1, 2, and 5), all of which resulted in recurrence of DHS within a few months. Eventually, all patients underwent long-segment posterior corrective fusion extending from the occiput or C2 to either T1 or T2.

Postoperatively, cervical kyphosis was corrected, and cervical lordosis was restored (Figure 2).

**Figure 2:** Postoperative neutral lateral cervical radiographs A: Case 1; B: Case 2; C: Case 3; D: Case 4; E: Case 5. Posterior fixation from the occiput or C2 to Th1/Th2 was performed. Cervical kyphosis was corrected in all cases. The numerical identifiers (e.g., Case 1, Case 2, Case 3, etc.) are arbitrary and were created solely for the purpose of referencing specific cases within this article. These identifiers do not correspond to any patient-identifying information.

The C2-C7 SVA improved to within the normal range, and the T1 slope was reduced. Four patients regained the ability to maintain horizontal gaze for more than 30 minutes, with marked improvements in clinical outcomes. In Case 3, although postoperative gaze maintenance was achieved, the patient developed aspiration pneumonia and died shortly before discharge.

Representative case: Case 1

A 69-year-old woman with no notable past medical history presented to our hospital with a chief complaint of progressive difficulty in maintaining forward gaze due to acute cervical flexion. Her symptoms gradually worsened, leading to impaired oral intake and gait disturbance.

At initial presentation, she was alert and exhibited no cranial nerve abnormalities. Although no apparent limb paralysis was observed, she demonstrated marked muscle weakness, numbness in both hands, and impaired fine motor skills. Deep tendon reflexes in all extremities were hyperactive, and both Hoffmann and Wartenberg signs were positive.

Cervical spine radiographs revealed kyphotic deformity (Figure 3A).

**Figure 3:** Preoperative Images A: Lateral plain radiograph showing cervical kyphosis; B: Cervical CT and C: MRI reveal local kyphosis at the C4–C6 levels with bony changes on the anterior vertebral bodies (arrows); D: Anteroposterior and posterior fixation was performed from C4 to C6.

CT and MRI in the extended neck position showed focal kyphosis from C4 to C6 (Figures 3B, 3C). Bony changes were noted at the anterior aspects of the C5 and C6 vertebral bodies (Figures 3B, 3C). Although mild dural sac compression was present, no significant spinal canal stenosis was observed (Figure 3C). Blood tests showed normal thyroid function and creatine kinase levels, with no other significant abnormalities on biochemical analysis.

The patient was diagnosed with DHS. Conservative treatment, including cervical collar support and manual interventions, failed to improve her condition, and progressive symptom deterioration was noted. Therefore, surgical intervention was planned. Anterior and posterior cervical fixation from C4 to C6 was performed (Figure 3D).

Postoperatively, her symptoms temporarily improved; however, two months later, recurrent cervical flexion was observed, and cage subsidence at the C5/C6 level was identified. As a result, an additional posterior fixation from the occiput to the thoracic spine was performed (Figure 4).

**Figure 4:** Intraoperative and postoperative images A: Intraoperative photograph showing occiput to T2 posterior fixation. The upper and lower ends of the rods are secured using Nesplon tape (arrows); B: Postoperative anteroposterior radiograph; C: Lateral radiograph demonstrating correction of cervical kyphosis following posterior fixation.

Pedicle screws were placed at C2, Th1, and Th2, and lateral mass screws at C3 through C6, supplemented with Nexlon tape reinforcement (Figure 4A).

Following the second surgery, the patient regained ambulatory function. At one year postoperatively, no recurrence of cervical flexion has been observed.

## Discussion

DHS is a condition characterized by marked forward flexion of the head due to dysfunction of the cervical extensor muscles, and it predominantly affects elderly women [1-4,6,7]. The etiology of DHS is diverse and can be anatomically classified into three major types: (1) localized cervical kyphosis, (2) thoracolumbar malalignment leading to forward flexion, and (3) a diffuse global kyphosis combining both features [6,13]. All cases in the present study were classified as the localized cervical type, with no thoracolumbar kyphosis.

The onset pattern of DHS varies among individuals and is generally categorized into two types: acute, which progresses rapidly within a few days, and chronic, which develops gradually over several months [11,14]. Endo et al. previously reported a case of acute-onset DHS [11], and our Case 1 similarly exhibited acute onset, with impaired horizontal gaze developing within three days. This patient had no concurrent neurological disorders, suggesting INEM as the sole etiology.

Common radiological findings in DHS include cervical kyphosis, cervical spondylolisthesis, and anterior deviation of the SVA [5,6,9,10]. The normal SVA of the cervical spine in Japanese individuals is approximately 20 mm, and according to the classification by Ames et al., deformity is defined using a threshold of 40-43 mm [5,9]. In our case series, SVA ranged from 32 to 70.7 mm, and the C2-C7 Cobb angles ranged from -3° to -49°, indicating pathological kyphosis in all patients. The T1 slope ranged from 11° to 43°, suggesting disrupted sagittal balance and abnormal cervical alignment. DHS is believed to result from a vicious cycle in which age-related weakening of the cervical extensors, degenerative changes in the upper cervical spine, and spondylolisthesis progress over time, leading to compensatory forward flexion due to neck pain and radiculopathy (e.g., numbness or clumsiness in the hands), which in turn exacerbates disuse atrophy of the extensor muscles [3,5-8].

Interestingly, in all cases in this study, the cervical kyphosis was relatively flexible, and intraoperative correction allowed realignment to a near-normal lordosis. A key distinction in DHS is whether the deformity is reversible (flexible) or fixed (rigid). Fixed deformities typically result from longstanding structural changes such as severe osteophyte formation, autofusion, or ankylosis, and often require more aggressive osteotomy procedures to achieve correction [3,4,12]. In contrast, reversible deformities are characterized by sagittal malalignment due primarily to muscle dysfunction or early-stage structural degeneration, where the cervical spine can be realigned without osteotomy [3,4]. Our cases predominantly exhibited reversible deformities, which allowed for successful realignment using long posterior fusion without the need for extensive bone resection. This highlights the importance of early identification of deformability in selecting an appropriate surgical strategy.

Conservative treatment, including whole-body muscle training and rehabilitation, is considered the first-line approach for DHS [14]. This is because the postural compensation caused by DHS extends beyond the cervical region, often involving thoracic kyphosis and knee flexion. Therefore, improving overall muscular function is more effective than local interventions. However, rehabilitation alone often takes more than six months to yield symptomatic improvement, and in cases of progressive DHS or severe impairment of ADL, timely surgical intervention is recommended [10,12,14].

In our cases, considering the patients were elderly females with osteoporosis, low invasiveness and instrumentation safety were prioritized. Initially, short-segment fusion combined with laminoplasty was performed in Cases 1, 2, and 5. However, all three experienced recurrence of DHS within a few months and exhibited disrupted sagittal alignment postoperatively. Previous studies have reported relatively high recurrence rates in patients undergoing short-segment fusion for DHS [12]. These findings highlight the inherent limitations of short-segment fusion in maintaining long-term sagittal alignment in vulnerable populations. In particular, patients with atrophic posterior cervical muscles on MRI were at high risk of postoperative cervical instability when treated with laminoplasty alone, necessitating careful surgical planning. Eventually, all patients underwent long-segment posterior corrective fusion extending from C2 or the occiput to T1 or T2, resulting in good realignment and improved clinical outcomes. Minimal corrective maneuvers were employed, and maintaining the natural corrective posture via long fusion proved effective in patients with flexible DHS. Long-segment constructs offer biomechanical advantages by distributing mechanical loads across a greater number of fixation points, thereby reducing stress on individual segments and minimizing the risk of implant failure. In osteoporotic patients, such constructs help prevent adjacent segment degeneration and junctional kyphosis, both of which are common complications following short fusion [3,4,12]. This extended support contributes to more durable sagittal alignment and improved functional outcomes. In most cases of DHS, long-segment posterior fixation extending from C2 to the upper thoracic spine is sufficient to achieve stable correction [3,4,12]. Occipitocervical fixation is generally reserved for cases involving craniovertebral instability, anatomical constraints such as severe degeneration at C1-C2, or compromised bone quality that precludes reliable instrumentation at C2 [12]. In our Case 1, however, occipitothoracic fusion was selected after recurrence occurred following a prior short-segment fusion. Although fixation from C2 might have been biomechanically sufficient in retrospect, we opted for a more extensive construct to ensure maximum stability and minimize the risk of a second failure. This decision was influenced by the patient’s history of recurrence, as well as the strong desire to restore horizontal gaze and functional posture definitively. We acknowledge that this may have resulted in overtreatment, but in select cases with a high risk of recurrence or poor anchoring at C2, occipital fixation may be justifiable.

The surgical method used involved posterior fixation from C2 to the upper thoracic spine using C2 pedicle screws and Nesplon tape (Alfresa Pharma Co., Ltd., Osaka, Japan). This approach was chosen to achieve both rigidity and flexibility, considering the high prevalence of osteoporosis in elderly women. Recent reports have shown that long-span fusion from the cervical to the thoracic spine reduces the risk of recurrence and contributes to maintaining horizontal gaze and improving quality of life [11], consistent with our favorable results.

These results suggest that long-segment corrective fixation not only improves radiological parameters but also translates into functional gains such as sustained horizontal gaze and better daily activity performance. However, clinicians should remain vigilant regarding postoperative systemic complications, especially in frail elderly patients. This highlights the importance of careful systemic management in elderly patients, even when surgical correction of DHS is successful.

In conclusion, surgical intervention, particularly long-segment corrective fusion, is an effective treatment option for DHS cases that are refractory to conservative therapy or exhibit reversible kyphosis. Detailed preoperative evaluation of sagittal alignment and the condition of the posterior cervical muscles is essential for selecting the appropriate surgical method and fusion range, thereby ensuring stable correction and high patient satisfaction.

This study has several limitations. First, it was a retrospective case series with a small sample size of five patients, all from a single institution, which may limit the generalizability of the findings. Second, although radiographic parameters were analyzed in detail, standardized pre- and postoperative functional assessments such as ADL scores or the Neck Disability Index were not uniformly available, restricting objective evaluation of clinical outcomes. Third, given the lack of long-term follow-up beyond one year in most cases, the durability of the surgical correction and the potential for delayed complications remain unclear. Lastly, surgical decision-making, including the extent of fixation, was individualized and not based on a standardized protocol, which may have introduced selection bias. Future prospective studies with larger cohorts and standardized outcome measures are warranted to validate the efficacy of long-segment fixation for DHS.

## Conclusions

In this report, we retrospectively analyzed five cases of DHS treated surgically at our institution. While short-segment fixation was insufficient to prevent recurrence in some cases, long-segment corrective fixation from C2 to the upper thoracic spine effectively improved cervical alignment and clinical outcomes.

Future studies with larger case series and longer follow-up periods are warranted to establish more definitive evidence regarding surgical indications and procedural selection in the treatment of DHS.
